The article "An Application of ITO Analysis in Secondary Kinship Identification" was published in 2022. Journal: Comput Math Methods Med.

# An Application of ITO Analysis in Secondary Kinship Identification

**DOI:** 10.1155/2022/4381979

**Published:** 2022-07-01

**Authors:** Peng Zhou, Xuemei Chen, Qianrong Wang, Junfu Wang, Xiaoqun Xu, Ran Wei

**Affiliations:** ^1^Shandong Provincial Hospital Affiliated to Shandong First Medical University, Jinan, China; ^2^School of Clinical and Basic Medical Sciences, Shandong First Medical University & Shandong Academy of Medical Sciences, Jinan, China; ^3^The Third Affiliated Hospital of Shandong First Medical University, Jinan, China

## Abstract

**Objective:**

As the methods of the paternity and kinship testing have been developed, the second-degree and more distant relationships remain challenging in forensic science. Currently, the ITO method is the mainstream method to clarify the kinship between two individuals.

**Methods:**

In this study, the ITO algorithm was used to calculate the uncle-nephew index based on 55 autosomal short tandem repeats (STRs) loci that were universally used for forensic identification. 19 STRs loci in Y chromosome were used for verification of the kinship.

**Results:**

The cumulative uncle-nephew index between A and B was calculated to 0.993 by the analysis of the genotyping results of 21 STRs. When genotyping results of the other 34 STRs were added to the calculation algorithm, the cumulative uncle-nephew index between A and B was promoted to 227.928. Meanwhile, genotyping results of 17 Y-STRs loci showed that A and B shared the same Y-STRs haplotype that was in accord with the paternal inheritance law.

**Conclusion:**

The biological uncle-nephew relationship between A and B are identified by applying the statistical principles and genetic technologies.

## 1. Introduction

In forensic genetics, short tandem repeats (STRs) on autosomes is the frequently-used genetic markers in the mainstream at present [1, 2]. The stochastic ITO transition matrices provided by Li and Sacks in 1954 is a traditional methods to obtain the joint STR genotype distribution and genotypic correlations between any specified pair of noninbred relatives [3, 4]. However, the sibling identification is complicated, and the conclusions risk uncertainties in some cases, because the potential intimate kinship between the two individuals involved in the kinship testing may limit the amount of genetic information that is usable for the identification. In this case study, an adult male (A) suspected that he might be abducted and trafficked into his current family at his early age. Because both the suspected father and the suspected mother died due to physical reasons and no material samples could be collected, the paternity identification could not be conducted. So the man (A) requested an identification of the uncle-nephew kinship with his alive suspicious uncle (B). We applied the ITO algorithm using STRs in autosomes and Y chromosome in the identification of this secondary kinship. The validity of the ITO algorithm will provide more reliable evidences for the kinship identification.

## 2. Materials and Methods

### 2.1. Sample Collection and DNA Extraction

Blood spot samples were taken from the fingertip of A and B. DNA samples were extracted by 5% Chelex-100 (Sigma-Aldrich, USA) extraction method.

### 2.2. PCR Amplification

55 pairs of primers for STRs on autosomes were obtained from SiFaSTRTM 23 Plex Identification System (China Academy of Forensic Science, China), GoldeneyeTM 22NC Identification System (Jidian Cognitive Technology Co., Ltd., Beijing, China), and AGCU 21+1 STR Fluorescence Detection kit (Zhongde Meilian Biotechnology Co., Ltd., Wuxi, China). 17 pairs of primers for Y STRs were obtained from Goldeneye DNA 27Y Identification System (Jidian Cognitive Technology Co., Ltd., Beijing, China). PCR reactions were performed according to the manual of each kit.

### 2.3. Capillary Electrophoresis and Genotyping Analysis

Capillary electrophoresis was performed using a 3130 XL Genetic Analyzer (Thermo Fisher Scientific, Waltham, MA, USA), and genotype detection and analysis were performed using GeneMapper ID-X software (Thermo Fisher Scientific, Waltham, MA, USA).

### 2.4. Statistical Analysis

The ITO method was applied to calculate the uncle-nephew index using genotyping data of 55 autosomal STRs loci, and the verification of the uncle-nephew kinship is carried using genotyping data of 17 Y-STRs loci.

## 3. Results

### 3.1. Genotyping of Autosomal STRs Loci

With the credible negative and positive quality controls, valid genotyping of total 55 STRs loci on autosomes in A and B was conducted. The genotyping results are shown in Table 1. A and B had different STRs on homologous chromosomes at 14 loci (vWA, D21S11, D18S51, D12S391, FGA, D15S659, D3S3045, D17S1290, D2S441, D11S2368, D7S3048, D5S2500, D4S2408, and D2S1776). At the other 41 loci, A and B shared at least one STR haploid. Among them, at 7 loci (D19S433, D13S317, D4S2366, D13S325, D6S474, D6S1017, and D9S1122), A and B shared the same genotype.

### 3.2. Genotyping of Y-STRs Loci

With the credible negative and positive quality controls, valid genotyping of total 17 Y-STRs loci in A and B was conducted. The genotyping results are shown in Table 2. A and B shared the same genotype on all the 17 Y-STR loci.

### 3.3. Calculation for the Uncle-Nephew Index

The uncle-nephew index is calculated using the formula W = PI/(PI + 1). The cumulative uncle-nephew index between A and B was calculated to 0.993 by the analysis of the genotyping results of 21 STRs (from SiFaSTRTM 23 plex identification system). This value was in the middle area that the uncle-nephew kinship could not be identified or excluded. When genotyping results of the other 34 STRs (from Goldeneye™ 22NC Identification System and AGCU 21+1 STR Fluorescence Detection kit) were added to the calculation algorithm [5], the cumulative uncle-nephew index between A and B was promoted to 227.928. The uncle-nephew index between individuals A and B was calculated as 21%, 40%, 69%, and 95% based on the genotyping data of 19, 29, 39, and 55 autosomal STRs separately. Meanwhile, genotyping results of 17 Y-STRs loci showed that A and B shared the same Y-STRs haplotype that was in accord with the paternal inheritance law. Therefore, based on the existing information and genetic analysis results, there is a high possibility that a biological uncle-nephew relationship between A and B exists.

## 4. Discussion

A complete description of the degree of relatedness of two individuals is a common and fundamental request in the forensic genetics [6]. In this case, there is an urgent demand for kinship identification without the genetic information of parents. However, there is no common standard for uncle-nephew kinship identification. So firstly, we used the genotyping results of 21 STRs from the conventional kit, SiFaSTRTM 23 plex identification system. The calculation method was revised according to the preliminary result, and the sufficient number of STRs loci was added. All STRs loci used in this study are all loci frequently used in forensic identification practice and have abundant population data which provide a reliable basis for the calculation reliability and the implementation feasibility. Meanwhile, when the uncle-nephew kinship was identified with relatively low index, the Y-STRs locus is a useful supplement in case that the tested individuals are all male [7]. The same Y-STRs haplotype found in the tested individuals enhance the reliability of the identification.

This study calculated the uncle-nephew index using ITO method [3]. The ITO method is a classic way to identify the kinship between two individuals. Shao et al. pointed out that after the conclusion that shared alleles cannot be excluded from the analysis, ITO method can be further used to establish discriminant assumptions according to the specific case to obtain objective and reliable identification opinions [8]. In our study, it is demonstrated that when more autosomal STRs were used, the more uncle-nephew index between individuals A and B was obtained. It is demonstrated that the accuracy rate of the uncle-nephew kinship identification between two individuals increases with the number of the genetic markers. Therefore, more loci should be genotyped within the maximum testing capacity of the forensic laboratory's capacity for the complex kinship identifications, such as uncle-nephew relationships. However, the sufficient number of genetic marker loci and the rage of the probability value to verify the kinship in the complex cases should be investigated.

With the development of high-throughput sequencing and the establishment of genome database, kinship testing based on multiple genetic markers, such as SNPs and microhaplotypes, has great valuable practical applications [9, 10]. In the future, we will apply more genetic markers, such as SNPs and indels, in solving complex kinship testing problems based on high-throughput sequencing [11, 12].

## Figures and Tables

**Table 1:** Genotyping of 55 autosomal STRs loci in A and B.

STRs locus	A	B
D3S1358	15, 19	14, 19
D5S818	10, 12	10, 13
D2S1338	23, 25	17, 25
TPOX	8, 9	8, 11
CSF1PO	10, 12	12, 12
Penta D	11, 13	9, 11
TH01	8, 9	7, 8
vWA	16, 17	14, 18
D7S820	11, 11	9, 11
D21S11	31.2, 31.2	30, 32
Penta E	12, 16	5, 12
D10S1248	13, 16	12, 13
D8S1179	14, 15	13, 14
D1S1656	17, 17	15, 17
D18S51	13, 14	16, 22
D12S391	19, 24	20, 23
D6S1043	12, 15	12, 20
D19S433	14, 14.2	14, 14.2
D16S539	9, 9	9, 12
D13S317	11, 13	11, 13
FGA	22, 26	23, 23
D4S2366	9, 12	11, 12
D6S477	15, 16	16, 17
D22-GATA198B05	20, 21	21, 21
D15S659	10, 12	15, 16
D8S1132	21, 21	21, 22
D3S3045	13, 13	11, 14
D14S608	10, 11	9, 10
D17S1290	11, 16	15, 15
D3S1744	17, 19	13, 19
D2S441	11, 12	13, 14
D18S535	10, 16	10, 12
D13S325	19, 20	19, 20
D7S1517	24, 25	23, 25
D10S1435	12, 12	11, 12
D11S2368	18, 20	19, 21
D19S253	13, 14	7, 13
D7S3048	24, 24	18, 21
D5S2500	9, 14	12, 16
D6S474	15, 15	15, 15
D12ATA63	16, 17	12, 17
D22S1045	15, 17	13, 17
D1S1677	14, 14	10, 14
D11S4463	14, 16	14, 14
D1S1627	13, 14	11, 14
D3S4529	13, 14	14, 15
D6S1017	8, 12	8, 12
D4S2408	9, 9	7, 10
D17S1301	12, 13	12, 12
D1GATA113	7, 7	7, 13
D18S853	11, 14	11, 11
D20S482	13, 13	13, 14
D14S1434	11, 14	12, 14
D9S1122	13, 13	13, 13
D2S1776	11, 12	9, 14

**Table 2:** Genotyping of 17 Y-STRs loci in A and B.

Y-STRs loci	A	B
DYS456	16	16
DYS389I	13	13
DYS390	23	23
DYS389II	29	29
DYS458	16	16
DYS19	14	14
DYS385a/b	13/14	13/14
DYS393	12	12
DYS391	10	10
DYS439	12	12
DYS635	21	21
DYS392	14	14
Y GATA H4	12	12
DYS437	15	15
DYS438	11	11
DYS448	20	20

## Data Availability

The experimental data used to support the findings of this study are available from the corresponding author upon request.
